# Efficacy and Safety of Chinese Medicine in Treating Arrhythmia: Meta-Analysis of Randomized Controlled Trials

**DOI:** 10.1155/2021/9960471

**Published:** 2021-10-29

**Authors:** Hanyu He, Guoning Han, Xinju Li, Hongyi Lan, Ying Li, Xiaoxin Dou, Yi Guo, Mingxing Zhang, Hongyan Liu

**Affiliations:** ^1^School of Traditional Chinese Medicine, Tianjin University of Traditional Chinese Medicine, Tianjin 301617, China; ^2^School of Acupuncture & Moxibustion and Tuina, Tianjin University of Traditional Chinese Medicine, Tianjin 301617, China; ^3^School of Integrative Medicine, Tianjin University of Traditional Chinese Medicine, Tianjin 301617, China

## Abstract

**Objective:**

To evaluate the clinical efficacy of traditional Chinese medicine in the treatment of arrhythmia.

**Methods:**

The researchers searched CNKI, VIP, WF, PubMed, Web of Science, and Cochrane Library with the set-up themes as randomized controlled trials (RCTs) on the clinical efficacy of traditional Chinese medicine in the treatment of arrhythmia. This research evaluated all the retrieve literature and conducted selection based on the evaluation. Stata software was applied for meta-analysis.

**Results:**

23 articles were retrieved with a total patient number of 2846. The results observed from the meta-analysis indicated the following: (1) compared with the result showed in placebo group, the traditional Chinese medicine group presented to have good efficacy, especially in the treatment of premature ventricular contractions. (2) In comparison with the western medicine group, the curative effect of Chinese medicine could approximately equal the therapeutic effect as western medicine. (3) Compared with the application of sole western medicine group, the combination of both traditional Chinese medicine and western medicine could have a better curative effect.

**Conclusion:**

In the treatment of arrhythmia disease, the application of traditional Chinese medicine can be considered as an effective method. In addition to that, the therapeutic effect obtained from the combination of both Chinese traditional medicine and western medicine is clinically better than that of the sole use of western medicine.

## 1. Introduction

Arrhythmia is a common disease of clinical cardiovascular, which can be divided into two types, namely, tachyarrhythmia and bradycardia. Tachyarrhythmia includes clinical symptoms, such as atrial fibrillation, atrial flutter, atrial tachycardia, ventricular tachycardia, ventricular fibrillation, atrial premature beat, and ventricular premature beat, and the second type of arrhythmia-bradycardia covers symptoms, such as sinus bradycardia, conduction block, and sick sinus syndrome. At present, the treatment of bradyarrhythmia with western medicine mainly includes two methods, namely, drug treatment and the implantation of artificial cardiac pacemaker. However, certain drugs did not show sufficient evidence for relevant efficacy, so it is difficult to promote these medicines for wild use [1], and, in the meantime, the cost for artificial pacemakers is too high to fully meet the clinical needs. Therefore, timely and effective prevention measures for arrhythmia and economic treatment are of important clinical significance.

The academic term for arrhythmia did not exist in the traditional Chinese medicine, but it can be classified in the disease as “Xinji (palpitations)” according to its clinical manifestations. Recent years have witnessed a great number of studies to prove that traditional Chinese medicine shows strengths in the prevention and treatment of arrhythmia in certain extent, and it could function to alleviate the rate of complications.

Before the researches showed hard evidence, Hu et al. [2] carried out a meta-analysis to study the treatment of bradyarrhythmia with Chinese patent medicine. However, this literature mainly studied four Chinese patent medicines, Shenxianshengmai oral liquid, Xinbao pill, Ningxinbao capsules, and Shensongyangxin capsules, and studied that the disease was bradyarrhythmia; Sun and Wang [3] further carried out a meta-analysis on the treatment of arrhythmia with traditional Chinese medicine decoction. However, the above two meta-analysis research studies only focused on one dosage form or a single disease, as for the scientific and effective grouping, they are not included in their study. Therefore, this article mainly collected all randomized controlled trials (RCTs) of traditional Chinese medicine (including Chinese patent medicine and decoction) on the relevant treatment of arrhythmia, adopted a more scientific and effective subgroup classification method, and conducted the meta-analysis on its clinical efficacy, in order to provide more scientific evidence for the clinical practice of Chinese traditional medicine.

## 2. Materials and Methods

### 2.1. Eligibility, Data Sources, and Searches

The randomized controlled trials (RCTs) with the application of Chinese medicine or the combination of traditional Chinese medicine with the conventional western medicine in the treatment of arrhythmia were retrieved in the study. The languages of documents were limited to Chinese and English. Patients who are diagnosed with arrhythmia shall meet the standards of the modern medical diagnosis criteria. The total effective rates with 24-hour Holter were used as the indexes of study.

The Chinese documents databases, such as CNKI, VIP, and WF, along with the English databases of documents, such as PubMed, Web of Science, and Cochrane Library, were retrieved by computer. Words, such as Chinese patent medicine, traditional Chinese medicine, Chinese and western medicine, arrhythmia, bradycardia, tachycardia, and palpitation, were selected and input as the keywords for retrieval. The retrieval time was from the establishment of the database to July 2020. Exclusion criteria were set as the following: (1) repeated published literature; (2) other heart diseases, unrelated to this study, news reports, treatment manuals, and conference papers; (3) animal experiments, reviews, theoretical literature, case reports, and data analysis; (4) non-Chinese medicine treatment literature, such as acupuncture and massage; (5) incomplete and confused data in the literature; (6) unclear random methods and inappropriate control groups; and (7) the improved Jadad score, which is lower than 4 points. The review is registered on PROSPERO, registration number CRD42020204479.

### 2.2. Data Selection

The repeated literature was searched by NoteExpress, and those repeated documents were selected out manually; according to the inclusion and exclusion criteria, the titles and abstracts of the searched documents were read for the purpose of selecting out those that obviously did not meet the inclusion criteria, and then the full text of the retrieved documents was obtained and further read to exclude those that did not meet the inclusion criteria or had obvious reasons for exclusion. The data of the included research studies were selected by the application of a predesigned data extraction table, which includes basic information of patients, baseline condition of patients' diseases, intervention and control measures, treatment course, and outcome indicators. In terms of disagreement, it shall be resolved through discussion or consultation by the presence of a third party.

### 2.3. Quality Assessment

In accordance with Cochrane Handbook 5.3, the method for bias risk assessment was used to serve the purpose of evaluating the bias risk of the included documents. Along with the random allocation method, this study mainly explored the the following factors: whether the allocation was hidden, blind method, the integrity of the results data, selective reporting of research results, and other sources of bias. Each evaluation result was divided into three levels based on their degree of risks: low risk, unclear, and high risk. In the meantime, the methodological quality of the selected studies was evaluated in accordance with the modified Jadad scale, which includes (1) random sequence generation: 2 points for suitable method, 1 point is for unclear, and 0 points for inappropriate; (2) hidden allocation: 2 points for suitable method, 1 point for unclear, and 0 points for inappropriate or not used; (3) blind method: 2 points for suitable method, 1 point for unclear, and 0 points for inappropriate; (4) withdrawal: 1 point for description and 0 points for zero description. The total score of the scale is 7.

### 2.4. Data Synthesis and Analysis

The data were analyzed by the Stata software. The procedure goes as follows. Firstly, the heterogeneity of clinical trials was determined by the heterogeneity test. If *P* ≥ 0.05, *I*^2^ ≤ 50%, it can be considered as homogeneity of multiple similar studies, and a fixed effect model is used for evaluation; if *P* < 0.05, *I*^2^ > 50%, it can be considered as heterogeneity of multiple studies. Then, the random effect model will be put into use for further conduction of meta-analysis. In this experiment, the ratio (RR) was used as the combined statistic.

## 3. Results

### 3.1. Database Review and Characteristics of Selected Documents

A total number of 6540 related documents were selected both automatically and manually, including 6136 in Chinese and 404 in English. After manually removing the repeated documents through scanning over the title and abstract, there are 679 papers remaining (including two English documents). Next, the full text is read and a qualitative and quantitative analysis is conducted on the literature. Last but not least, 23 articles (including one English document) [4–26] were included. The search process is shown in Figure 1.

The following literature was excluded. (1) There were 1019 repetitive articles. (2) There were 3363 papers on other heart diseases, unrelated to this study, news reports, treatment manuals, and conference papers. (3) There were 1143 articles on animal experiments, reviews, theoretical literature, case reports, and data analysis. (4) There were 108 papers on acupuncture and massage. (5) There were 885 literatures with unclear random methods and inappropriate control groups. (6) There were 28 articles with inappropriate outcome indicators. (7) There were 17 articles with improved Jadad score <4.

23 RCTs were included in this study; every one of them goes through double-blind test, with a total number of 2846 patients, which includes 1517 cases in the experimental group and 1329 cases in the control group, and the single study sample size is 20–292 cases. The intervention measures took in the treatment, which are involved in the study, included Tongmai Yangxin pill, Xinbao pill, Zengsheng Fumai decoction, Shensong Yangxin capsule, fulvning granule, Jiawei Ningxin Decoction, Jiawei Shengmai San, kuailuning, Ningxin Changmai drink, Huxin recipe, Ningji granule, Xinzhenning pill, Xinning capsule, Yangyin Xifeng decoction, Yiqi Fumai Granule, Yiqi Yangyin formula, and Yiqi Yangxin gum Bursa. The basic characteristics of the included documents are shown in Table 1.

### 3.2. Evidence of Grading Quality

The risk assessment of bias in the included documents is shown in Figure 2.

### 3.3. Main Results

The difference between the abovementioned two groups was shown in comparison by the forest map, and the RR value was compared as well. The total effective cases in the experimental group and the control group were 1131/1517 and 700/1329, respectively, and the correlation index value of heterogeneity test was *I*^2^ = 73.1%, *P* < 0.05; hence, the fixed effect model was applied. The combined RR value was 1.37 (1.23, 1.53) and *P* < 0.05, which indicates that a significant difference exists in the clinical effective rates between the experimental group and the control group (Figure 3).

In regard to the 23 documents in the single study sample, 8 were focused on the comparative study with placebo, 8 documents emphasized the comparative study between Chinese medicine and western medicine, and 7 aimed to study the differences among the traditional Chinese medicine and western medicine, as well as conventional western medicine. The 23 documents were divided into three subgroups for comparative analysis.

#### 3.3.1. Compared with Placebo

The difference between the two groups was compared with the assistance of forest map, and the RR value was compared as well. The correlation index of heterogeneity test was *I*^2^ = 89.6%, *P* < 0.05, so the fixed effect model was applied. The combined RR value was 2.16 (1.3, 3.6), *P* < 0.05, which indicates that the clinical effective rates of the experimental group and the control group were significantly different. Among them, 2 articles were focused on the treatment of premature ventricular contractions, 5 articles studied the treatment of bradyarrhythmia, and 1 article explored the treatment of premature contractions. Because of the existence of heterogeneity, the analysis of subgroups was performed twice in accordance with the disease type (Figure 4).

The ventricular premature beat group was observed to have *I*^2^ = 0.0%, *P*=0.962 > 0.05, which proves the consistency of the results, and the RR value was 2.78 (1.78, 4.34), *P* < 0.05, which suggests that the clinical effective rate of the experimental group was significantly different from that of the control group.

In the bradyarrhythmia group, the data obtained was *I*^2^ = 93.4%, *P* ≤ 0.01, which indicates the heterogeneity of the results, and the RR value was 2.50 (1.04, 6.00), *P* < 0.05, referring the existence of significantly difference between experimental group and control group in terms of the clinical effective rate. Among the selected articles, 2 articles were focused on the treatment with Zengsheng Fumai decoction, 2 articles were exploring the treatment with Xinbao pill, and the other one was the analysis of treatment with Shensong Yangxin capsule. Therefore, in accordance with the type of medication, subgroup analysis for the bradyarrhythmia group was conducted again (Figure 5). In the Zengsheng Fumai decoction group, *I*^2^ = 58.7%, *P*=0.120 > 0.05, indicating the consistency of the results, and the RR value is 1.29 (0.74, 2.25), *P* > 0.05, which suggests that no obvious difference was observed between the experimental group and the control group in terms of clinical efficiency. In the Shensong Yangxin capsule group, the RR value was 5.79 (3.14, 10.67), *P* < 0.05, which suggests that the clinical effective rate of the experimental group was significantly different from that of the control group. In the Xinbao pill group, *I*^2^ = 97.7%, *P* ≤ 0.01, which refers to the heterogeneity of the results, and the RR value was 4.46 (0.05, 433.63), *P* > 0.05, which means in regard to clinical efficiency, no significant differences were observed between the experimental group and the control group. For the heterogeneity analysis, Wei Dongfeng applied the method of the cross control, and Liu Yanxia adopted the method of random grouping control. Due to the difference of methods, there is a process of exchange between the treatment group and the control group in the clinical experiment of Weidongfeng, which leads to the difference of treatment baseline and forms heterogeneity with experiments of Liu Yanxia. Therefore, different baseline of treatment is resulted from the source of heterogeneity.

In the premature contraction group, the RR value reached 1.03 (0.79, 1.34), *P* > 0.05, which suggests that no significant difference in the clinical effective rate was observed between the experimental group and the control group.

#### 3.3.2. Compared with Western Medicine

Upon the comparative study of the difference between the two groups by forest map, the RR values were also compared to make a conclusion. The correlation index of heterogeneity test reached *I*^2^ = 0.0%, *P*=0.587 > 0.05. The combined RR value was 1.19 (1.11, 1.28), *P* < 0.05, which indicates the significant difference was observed in terms of the clinical effective rate between the experimental group and the control group. Among the documents of this group, 5 articles were studying the ventricular premature beat, 2 articles were studying the treatment of tachyarrhythmia, and 1 article was exploring the treatment for atrial fibrillation. In order to further explore the efficacy of traditional Chinese medicine in various diseases, subgroup analysis was conducted again in accordance with the disease types (Figure 6).

Through the observation of the ventricular premature beat group, values were shown as follows: *I*^2^ = 6.8%, *P*=0.399 > 0.05, which indicates that the results presented were featured by consistency, and the RR value was 1.18 (1.06, 1.30), *P* < 0.05, which suggests the existence of significant difference of clinical effective rate between the experimental group and the control group. Among the studied articles, 2 articles focused on the application of fumaining granules in the treatment, other documents focused on the use of Kuailuning capsule, Huxin formula, and Yangyin Xifeng Fumai decoction in the treatment. The subgroup analysis was further carried out in accordance with the specific medication situation (Figure 7). In fumaining granule group, *I*^2^ = 0.0%, *P*=0.628 > 0.05, which means the results obtained have consistency. The RR value was 0.87 (0.60, 1.28), *P* > 0.05, which means no obvious or significant differences were observed in terms of clinical efficiency between the experimental group and the control group. The RR values for Kuailuning Capsules and Huxin Recipe, respectively, were 1.23 (1.07, 1.43) and 1.26 (1.02, 1.55), *P* < 0.05, which means that the clinical effective rate of the experimental group was significantly different from that of the control group. The RR values of Yangyin Xifeng decoction was 1.09 (0.88, 1.36), *P* > 0.05, representing that there was no significant difference observed in clinical efficiency between the experimental group and the control group.

In the tachyarrhythmia group, the value obtained as the following was *I*^2^ = 6.8%, *P*=0.300 > 0.05, which means the results have consistency, and the RR value was 1.19 (1.06, 1.32), *P* < 0.05, which means that the clinical effective rate of the experimental group has significant difference with that of the control group.

In AF group, the RR value was 1.29 (1.02, 1.62), *P* < 0.05, suggesting the significant difference exists in terms of clinical effective rate between the experimental group and the control group.

#### 3.3.3. Traditional Chinese Medicine Combined with Western Medicine

This article detailed compared the difference between the two groups with the assistance of forest map and also conducted comparative study on the RR value. The correlation index of heterogeneity test was *I*^2^ = 0.0%, while *P*=0.920 > 0.05. The combined RR was 1.41 (1.30, 1.53), *P* < 0.05; the abovementioned data indicates that the clinical effective rate of the experimental group was significantly different from that of the control group. Among the studied groups, 4 articles were focused on the treatment of ventricular premature beat, 2 articles centered on the treatment of tachyarrhythmia and 1 article emphasize the treatment of atrial premature beat. In order to further explore the efficacy that traditional Chinese medicine has in various diseases, subgroup analysis was conducted again on the basis of the disease types (Figure 8).

In the ventricular premature beat group, *I*^2^ = 0.0%, *P*=0.720 > 0.05, which means the results obtained are consistent, and the RR value was 1.44 (1.31, 1.60), *P* < 0.05, which suggests that the clinical effective rate of the experimental group was significantly different from that of the control group.

In the analysis of tachyarrhythmia group, *I*^2^ = 0.0%, *P*=0.938 > 0.05, where we can conclude that the results are of consistency, and the RR value was 1.35 (1.13, 1.61), *P* < 0.05, which means the clinical effective rate didn't show significant difference between the experimental group and the control group.

In the atrial premature beat group, the RR value was 1.35 (1.05, 1.74), *P* > 0.05, which indicated that no significant difference was observed in clinical effective rate between the experimental group and the control group.

### 3.4. Safety Analysis

In regard to the 23 selected documents, 5 articles noticed the adverse reactions and reported the specific conditions of adverse reactions. Among them, 4 articles recorded the exact adverse reactions symptoms after taking traditional Chinese medicine, most of the adverse reactions were gastrointestinal reactions and dizziness, and the rate for the adverse reactions in the control group was observed to be higher than that in the experimental group. The remaining article recorded the adverse reactions of the control group. More details were shown in Table 2.

## 4. Discussion

The study conducted meta-analysis on the efficacy of traditional Chinese medicine in the treatment of arrhythmia. From the results obtained, it can be concluded that there are three main characters in the subgroups in terms of total. (1) In comparison with the placebo group, the traditional Chinese medicine group presented to have good curative effect in general, particularly in the treatment of ventricular premature beat. (2) In the comparative study with the western medicine group, the curative effect of traditional Chinese medicine can basically reach a similar therapeutic level as western medicine. In the treatment of tachyarrhythmia, VPB, and atrial fibrillation, certain traditional Chinese medicines show better curative effects compared with that of western medicines. (3) Compared with the solely application of the western medicine group in treatment, the combination of both traditional Chinese medicine and western medicine can achieve a better curative effect.

In respective analysis for subgroups, in the traditional Chinese medicine group and the placebo group, Yiqi Fumai granule, and Shensong Yangxin capsule do pose certain curative effect on the treatment of ventricular premature beat; Shensong Yangxin capsule shows a definite effect on the treatment of chronic arrhythmia. In comparison with western medicine group, traditional Chinese medicine (Xinning capsule, Xinjining pill) is considered to have better efficacy than traditional western medicine (propafenone and metoprolol tartrate) in terms of the control ability of tachyarrhythmia; in the treatment of ventricular premature beat, the curative effect that Chinese medicine Kuailuning capsule and Huxin prescription have has a better efficacy compared with that of western medicine group. However, as for the curative effect of fumaining granule, Yangyin Xifeng Fumai decoction is similar to that of western medicine group. In the treatment of paroxysmal atrial fibrillation, Jiawei Ningxin decoction is considered to be more efficient than amiodarone; in the control ability of premature contraction, the curative effect of Suanzaoren decoction is in a similar level compared with that of metoprolol succinate tablets. The combined application of both traditional Chinese medicine and western medicine in the treatment of ventricular premature beat, tachyarrhythmia, and atrial premature beat is believed to be better than the sole use of conventional western medicine (propafenone and metoprolol tartrate).

The study also contains certain deficiencies and limits. (1) Due to the complexity of the diseases that have been covered in this study, only the total effective rate of dynamic electrocardiogram was selected as the outcome index, which may not be able to comprehensively cover and evaluate the overall treatment effect. (2) This study mentioned various kinds of Chinese medicine intervention, and they may have certain differences in the curative effect, and some errors may also happen during the combined application of those medicines. (3) Some Chinese medicine groups only contain one group; therefore, it is difficult to highlight the group's effective effect. (4) Traditional Chinese medicine tends to treat the overall symptoms and alleviate the complications happening in human body, which might ignore the improvement of certain specific indicators. Therefore, even though some traditional Chinese medicines, which are selected in this study, may have failed to present therapeutic effect, they still have relevant relationship with the selected outcome indicators. (5) Some documents selected in this study only cover a small number of patients, which may cause certain errors.

To sum up, the results that obtained in this study show that in the treatment of arrhythmia disease, Chinese medicine can be considered as effective and could reach the similar treatment level as western medicine, and the therapeutic effect that the combined application of both Chinese and western medicine has is better compared with the simple use of western medicine in treatment. Therefore, in the clinical practice of arrhythmia, the therapeutic effect of traditional Chinese medicine on diseases can be considered, so as to adopt the treatment method of combined application of traditional Chinese medicine and western medicine. The use of traditional Chinese medicine for patients with either short-term or long-term treatment intervention can achieve the desired therapeutic effect. The quality of the literature included in this study is believed to be high for it contains a small degree of heterogeneity, the quality of methodology is acceptable, and the obtained results are of strong credibility and clinical significance. However, this study also has some common problems, which need to be verified by more high-quality, large sample, multicentered, long-term followup studies.

## Figures and Tables

**Figure 1:** Flowchart of included and excluded reports.

**Figure 2:** Assessment of quality of RCTs.

**Figure 3:** Forest plot and meta-analysis of TCM's effects on arrhythmia.

**Figure 4:** Forest plot and meta-analysis of TCM compared with placebo.

**Figure 5:** Forest plot and meta-analysis of different drugs' effect on bradycardia.

**Figure 6:** Forest plot and meta-analysis of TCM compared with western medicine.

**Figure 7:** Forest plot and meta-analysis of different drugs' effect on ventricular premature beat.

**Figure 8:** Forest plot and meta-analysis of TCM compared with TCM combined with western medicine.

**Table 1:** Characteristics of the included studies.

First author and year	Number of patients		Gender		Age (years)		Course of disease (year)		Study drug		Course of treatment (week)	Improved Jadad score	The type of disease
	Experimental	Control	Male	Female	Experimental	Control	Experimental	Control	Experimental	Control			
Yao 2006	137	134	153	149	47.0 ± 11.9	44.5 ± 11.7	6.8 ± 2.6	6.4 ± 2.4	Kuailuning capsules + placebo	Propafenone + placebo	12	7	VPB (ventricular premature beat)
Sun 2007	120	60	93	87	54.3 ± 9.4	53.4 ± 8.7	5.6	5.3	Xinning capsule	Propafenone	4	4	Tachyarrhythmia
Chen 2009	40	40	30	50	—	—	—	—	Shensong Yangxin capsules	Placebo	8	4	VPB
Sun 2011	24	20	16	28	63.6 ± 10.0	64.3 ± 5.9	—	—	Zengrate Fumai decoction	Placebo	3	4	Bradycardia
Chen 2012	43	43	28	58	65.0 ± 10.4	64.8 ± 6.3	—	—	Zengrate Fumai decoction	Placebo	3	5	Bradycardia
Li 2013	60	60	71	49	56.4 ± 9.2	55.8 ± 8.6	—	—	Yiqi Yangxin capsule + metoprolol tartrate tablets	Placebo + metoprolol tartrate tablets	8	4	VPB
Yu 2013	45	45	42	48	52.6 ± 10.7	51.3 ± 8.2	—	—	Fuluning granules + placebo	Propafenone + placebo	4	6	VPB
Liu 2014	115	104	107	112	—	—	—	—	Shensong Yangxin capsules	Placebo	4	7	Bradycardia
Guo 2015	23	21	18	26	54.1 ± 0.2	55.6 ± 12.0	—	—	Yiqi Fumai granules	Placebo	4	6	VPB
Liu 2015	30	30	25	35	50.5 ± 13.8	50.2 ± 11.3	2.7 ± 1.0	2.8 ± 1.1	Fuluning granules + placebo	Propafenone + placebo	4	5	VPB
Wei 2015	40	40	43	37	—	—	—	—	Xinbao pill	Placebo	12	4	Bradycardia
Li 2016	33	32	42	33	61.2 ± 8.7	61.3 ± 8.0	—	—	Tongmai Yangxin pill + metoprolol tartrate tablets	Placebo + metoprolol tartrate tablets	8	4	VPB
Yin 2016	174	68	118	124	54.1 ± 11.8	52.3 ± 12.2	—	—	Tongmai Yangxin pill	Placebo	4	4	Premature contraction
Hou 2018	30	30	29	31	60.1 ± 14.0	62.9 ± 11.7	1.6 ± 1.6	2.0 ± 1.6	Ning Tiao granule + metoprolol tartrate tablets	Placebo + Metoprolol Tartrate Tablets	4	5	Tachyarrhythmia
Wang 2018	31	31	32	30	58.1 ± 13.6	53.7 ± 15.5	1.2 ± 0.8	1.1 ± 0.7	Yiqi Yangyin recipe + metoprolol tartrate tablets	Placebo + Metoprolol Tartrate Tablets	12	5	VPB
Liu 2018	23	23	28	18	79.2 ± 5.1	81.3 ± 4.4	—	—	Xinbao pill	Placebo	12	4	Bradycardia
Sun 2019	292	292	273	311	56.2 ± 12.5	56.8 ± 12.0	—	—	Tongmai Yangxin pill + metoprolol tartrate tablets	Placebo + Metoprolol Tartrate Tablets	8	5	VPB
Xie 2014	32	31	34	29	—	—	—	—	Xin Jining pill	Metoprolol Tartrate Tablets	4	4	Tachyarrhythmia
Zhao 2016	50	50	56	44	59.1 ± 14.3	59.3 ± 15.5	4.6 ± 2.9	4.4 ± 2.0	HuxinJ recipe	Metoprolol Tartrate Tablets	4	4	VPB
Zhang 2017	69	68	65	72	56.1 ± 3.3	55.9 ± 3.0	—	—	Yangyin Xifeng Fumai decoction	Metoprolol	4	4	VPB
Yang 2017	35	30	33	32	55.8 ± 6.5	57.0 ± 6.5	—	—	Jiawei Ningxin decoction	Amiodarone	24	4	Atrial fibrillation
Chang 2018	29	31	24	26	59.6 ± 12.0	61.2 ± 10.5	—	—	Jiawei Shengmai San + conventional treatment	Conventional treatment	4	4	Tachyarrhythmia
Zhang 2019	45	48	50	43	59.4 ± 6.1	56.7 ± 7.3	3.2 ± 1.7	3.6 ± 1.8	Ningxin Changmai drink + metoprolol succinate	Metoprolol succinate	4	4	Atrial premature contraction

**Table 2:** Adverse reactions.

First author and year	Experimental/control									
	Number of samples	Gastrointestinal reactions	Av conduction block	Dizziness	Hypodynamia	Dry mouth	Hypotension	Insomnia	Sinus bradycardia	Elevated alt
Yao 2006	137\134	7/18	0/2	2/11	0/2	—	—	—	0/3	—
Wei 2015	40/40	6/4	—	—	—	4/0	—	—	—	—
Zhao 2016	50/50	0/3	—	1/4	—	—	1/0	—	—	—
Yang 2017	35/30	—	—	—	—	—	—	—	0/3	0/2
Wang 2018	31/31	2/5	—	1/2	0/1	—	1/1	0/3	—	—

## Data Availability

The raw data used to support the findings of this study are available from the first author upon request.
